This article has been retracted.

# The Research on the High-Protein Low-Calorie Food Recipe for Teenager Gymnastics Athletes

**DOI:** 10.2174/1874120701509010240

**Published:** 2015-08-31

**Authors:** Cong Wei

**Affiliations:** Dalian University, Dalian, China

**Keywords:** Gymnastics athletes, high-protein, low-calorie, teenager.

## Abstract

In order to prevent teenager gymnastics athletes getting fat deposition, weight gain, they should supply a rational food. This paper considers the normal growth and development of athletes, body fat deposition proteins and hunger feel, configured high-protein low-calorie food recipe. Then analysis the composition and the essential amino acids of the recipe. In the final choiced 18 adolescent gymnastics athletes as subjects, to verify the validity of the formula. And analysis the experimental results. The experimental results analysis shows that this recipe basically meets the design requirements.

## 1. INTRODUCTION

Protein refers to the level of the protein content of foods. Protein accounts for 16.3% of body weight. If exceeded, is called protein [1]. Animal protein with high protein is protein-rich foods, such as meat, poultry, fish and seafood. But the composition proportion of essential amino acids are close to the body needs, or containing high fat, cholesterol, is not well utilized by the body. Eatting high protein foods (as shown in Table **1**) can cause high cholesterol, and affect life expectancy [2].

## 1.1 Low-calorie Foods are Rich in Protein and Dietary Fiber, but Low in Calories

Gymnastics athletes need to maintain a beautiful lightweight body, to help complete a variety of skill moves [3]. In order to prevent athletes fat deposition, weight gain, it should supply a rational food [3]. This food can satisfy the needs of the body for a variety of nutrients, but also to reduce hunger and are not likely to cause fat deposition, should also be in line with our athletes' diet, which is the purpose of this study.

The rest of the paper is organized as follows. In Section 2, high-protein food and low-calorie food are summarized briefly. In Section 3, the food recipe is maded. In Section 4, experiments are presented and the results are discussed. Finally, a conclusion is provided in Section 5.

## 2. HIGH-PROTEIN FOOD AND LOW-CALORIE FOOD

Protein is an important material constituting the human body [6]. Various tissues (muscle, bone, skin, nerves) in body all contain protein. 

The material basis of growth is a protein. Therefore, the lean people gaining weight should eat more foods with protein-rich [4].

Low-calorie foods are rich in protein and dietary fiber, but low in calories. Here to introduce to you 10 low-calorie foods.

(1) **Almonds and nuts**: Nuts are rich in protein, fiber and a lot of trace elements and is very easy to have a sense of satiety. At 10:00 am and 15:00 pm, eat moderation nuts, that addresses your hunger, but also add energy.

(2) **Beans**: Beans are rich in dietary fiber, can absorb body moisture, but also to break down fat and inhibit fat accumulation, which will help purge. In addition, beans calories come from carbohydrates and high-quality soy protein [5].

(3) **Green vegetables**: Green vegetables are an important source of vitamins, minerals (calcium, phosphorus, potassium, magnesium, iron), dietary fiber and natural antioxidants [6].

(4) **Dairy products**: Dairy products rich in calcium species can promote bone growth. And a large number of high-quality protein can speed up your metabolism, so you burn more fat.

(5) **Oatmeal**: Oatmeal contains large amounts of dietary fiber, easy to produce satiety, promote metabolism. Let you burn more energy during digestion.

(6) **Egg**: Eggs are rich in high quality protein, essential amino acids the human body, vitamins and other trace elements potassium, sodium, magnesium and phosphorus. An egg has only 80 calories card.

(7) **Chicken and other lean meat**: Meat protein is the core of a variety of nutrients the human body needs. The normal human hormone secretion, the normal muscle growth and the normal immune system can not do without it [7].

(8) **Peanut Butter**: Peanuts are a good detoxification share, can strong intestinal, eliminate constipation. Phytic acid, plant sterols and other special materials in peanuts unique can increase the toughness of the intestine.

(9) **Olive oil**: Olive oil is rich in unsaturated fatty acids and vitamin E, can promote blood circulation and skin metabolism, stimulate digestion, lower cholesterol, relieve stomach pain, flatulence.

(10) **Whole wheat or cereal staple food**: Cereals are rich in dietary fiber, slow digestion in the human body, is also relatively low glycemic index [8].

### 2.1 Data Processing Method

In mathematics, mean has several different definitions depending on the context.

In probability and statistics, mean and expected value are used synonymously to refer to one measure of the central tendency either of a probability distribution or of the random variable characterized by that distribution. In the case of a discrete probability distribution of a random variable X, the mean is equal to the sum over every possible value weighted by the probability of that value。

(1) μ=∑xP(x)

In statistics, the standard deviation (SD) (represented by the Greek letter sigma, σ) is a measure that is used to quantify the amount of variation or dispersion of a set of data values.

Let X be a random variable with mean value μ:

(2) E[X]=μ

In the case where X takes random values from a finite data set x1, x2, ..., xN, with each value having the same probability, the standard deviation is

(3) $$\sigma =\sqrt{\frac{1}{N}\sum_{i=1}^{N}{\left(x_{i}-\mu \right)}^{2}}$$

Where $\mu =\frac{1}{N}\sum_{i=1}^{N}x_{i}$

### 2.2 Determine the Food Recipe

Gymnastics athletes need to maintain a beautiful lightweight body, to help complete a variety of skill moves. In order to prevent athletes fat deposition, weight gain, it should supply a rational food [9, 10]. 

This food can satisfy the needs of the body for a variety of nutrients, but also to reduce hunger and are not likely to cause fat deposition, should also be in line with our athletes' diet, which is the purpose of this study.

Fat deposition is due to the calories intaken faster than the body consumption. In a variety of nutrients, fat produces the most prolific calories. Excessive sugar intake is also easily transformed into fat. Heat productions of proteins is the same with carbohydrates, but not easily converted into fat, and has large dynamic action. So in recipe should minimize the content of fat and sugar, increase protein.

One of the keys to this recipe is a good selection of high-quality and taste vegetable protein. By comparison, it is determined to use the defatted peanut flour, mixed with wheat flour, cheese powder and whole egg, to produce amino acids complementary role.

Hunger is related to gastric emptying. Stomach filling something can inhibit the excitability of the central food, and hunger will be weakened. So recipe should contain no calorie filler. Konjac flour is a natural hybrid polysaccharides not digested and absorbed in the digestive tract, and has a strong swelling properties, good taste, easy processing and no bad taste. So we choosed konjac flour.

In order to maintain normal growth and development of athletes, should fortife iron, zinc and B vitamins in the formulation.

## 3. RECIPE EXPERIMENTAL ANALYSIS 

### 3.1 Analysis of Nutrients Concentration

The recipe was baked ans moistured removal. Use the Kjeldahl method to analysis protein (as shown in Fig. (**1**)). Use Soxhlet mention fat method to measure fat content. Carbohydrates are calculated after subtracting the crude fiber. The results are shown in Table **2**. From Table **2**, the sugar and fat content of the recipe was significantly less than in the general food, and protein content is high.

### 3.2 Analysis of Essential Amino Acids

Protein quality will depend on the type, the number and the proportion of essential amino acids, as shown in Fig. (**2**). Amino acids were analyzed by high performance liquid chromatography. The results are shown in Table **3**. Table **3** illustrates that the essential amino acid content of the formulation is rich, and full range, where the ratio would be more appropriate, much better than wheat flour, close to eggs.

### 3.3 The Trial Results of Gymnasts

In order to observe the effects of the athletes after consuming the recipe, we selected 18 teenager's gymnastics (male 10, female 8) from Wuhan Institute of Physical, and they were randomly divided into two groups. The control group did for ordinary diet, and the staple food of the experimental group was high-protein low-calorie recipe food. But the staple food calories of two were the same. Fruits and other non-staple food of two groups were basically the same. The experiment lasted 21 days. 

See Table **4** and Fig. (**3**), before and after the experiments the above indicators no significant changes. Urinary nitrogen content in the experimental group added 1.56g. Urinary nitrogen level represents the amount of decomposition of body protein. In the same weight, it simply reflects the ingestion of protein. This suggests that the experimental group was more than 7g of protein per day, which is equivalent to the protein content of 60 grams flour or an egg.

## CONCLUSION

In order to prevent teenager gymnastics athletes getting fat deposition, weight gain, they should supply a rational food. This paper considers the normal growth and development of athletes, body fat deposition proteins and hunger feel, configured high-protein low-calorie food recipe. Then analysis the composition and the essential amino acids of the recipe. In the final choiced 18 adolescent gymnastics athletes as subjects, to verify the validity of the formula. And analysis the experimental results. The experimental results analysis shows that this recipe basically meets the design requirements.

## Figures and Tables

**Fig. (1):** The nutrients concentration proportion.

**Fig. (2):** The composition of essential amino acids.

**Fig. (3):** The gymnastics athletes indicators before and after experiment.

**Table 1.** List of common high protein foods (protein content per 100 grams food).

Food	Concentration (g)	Food	Concentration (g)	Food	Concentration (g)
Oat	15.6	Lotus seeds	16.6	Dried mushroom	38.0
Lin Ma	21.9	Hazelnut	15.9	Peanut	26.2
Soy	36.3	Watermelon seed	31.8	Walnuts	15.4
Green beans	23.8	Pumpkin seeds	35.1	Pine nuts	16.7
Cowpea	22.3	Sunflower	23.1	Pigskin	26.4
Broad bean	28.2	Pork (lean)	16.7	Pig blood	18.9
Peas	24.6	Pig heart	19.1	Beef (lean)	20.3
Con	30.7	Liver	21.3	Lamb (lean)	17.3
Bean Curd	50.5	Pig kidneys	15.5		

**Table 2.** The nutrients concentration in the food recipe.

Nutrients	Concentration (g/100g)
Lipids	6.2
Protein	30.4
Carbohydrates	41.3
Other	22.1

**Table 3.** The composition of essential amino acids.

Amino acids	Concentration (mg/100g)
Lysine	1202
Methionine	351
Tryptophan	220
Threonine	765
Valine	1008
Leucine	1643

**Table 4.** Gymnastics athletes indicators before and after experiment.

Gymnastics athletes indicators	Control group		Experiment group	
	Before experiment	After experiment	Before experiment	After experiment
Height (m)	1.34±0.04	1.34±0.06	1.35±0.07	1.35±0.06
Weight (kg)	35.78±4.51	36.24±3.85	36.10±3.71	36.56±4.28
Uretic nitrogen (g/d)	10.25±0.38	10.28±0.45	10.68±0.31	12.24±0.39
Hb (g/L)	138.12±12.17	137.56±14.50	139.27±14.16	138.82±13.32
